This article has been retracted.

# Effects of Modified Sang ju-Yin Decoction Combined with IFN*α*lb Nebulization on IL-1*β* and HBD2 in Children with Asthmatic Bronchitis

**DOI:** 10.1155/2022/2802636

**Published:** 2022-06-22

**Authors:** Jun Zhang, You lan Wang, Ying ting Liu, Min Yuan, Jian guo Jin

**Affiliations:** ^1^Department of Child Healthcare, Wuhan Wuchang Hospital, Wuchang Hospital Affiliated to Wuhan University of Science and Technology, China; ^2^Pediatrics Department, Wuhan Yaxin General Hospital, China; ^3^Pediatrics Department of Xiantao First People's Hospital Affiliated to Yangtze University, China

## Abstract

**Background:**

Breathing disease swelling of the lung tubes caused by viral infection is more and more likely to develop into related to the lung tubes breathing disease, especially repeating breathing loudly.

**Objective:**

To investigate the effect of modified Sang ju-Yin Decoction combined with Interferon (IFN)*α*lb nebulization on children with asthmatic bronchitis and the effects of IL-1*β* and *β*-defensin 2 (HBD2).

**Materials and Methods:**

The clinical data of 80 children with asthmatic bronchitis who were diagnosed and treated in our hospital from May 2019 to May 2021 were selected as the research objects and divided into the control group and the observation group with 40 cases in each group according to different treatment methods. Among them, the control group was nebulized with IFN*α*lb, and the observation group was given addition and subtraction of Sang ju-Yin Decoction based on the control group. The clinical symptoms, pulmonary function indexes, adverse reactions, and effects on serum inflammatory indexes were observed and compared between the two groups.

**Results:**

There was no significant difference in the scores of symptoms and signs between the two groups before treatment (*P* > 0.05), while the scores of shortness of breath, cough, stridor, lung rales, and signs after treatment of observation group were better than those of the control group (*P* < 0.05). There was no significant difference in serum inflammatory indexes and pulmonary function indexes between the two groups before treatment (*P* > 0.05), while the differences in IL-6, IL-10, TNF-*α*, IL-1*β*, and HBD2 after treatment were significant between the two groups (*P* < 0.05). After treatment, the RR, TV, and PEF indexes of the two groups of children were significantly improved (*P* < 0.05). After treatment, the adverse reaction rate of liver function damage, dry throat discomfort, rash, nausea, and vomiting in the observation group was 7.5%, which was significantly lower than 27.5% in the control group (*P* < 0.05).

**Conclusion:**

Modified Sang ju-Yin Decoction combined with IFN*α*lb nebulization can improve symptoms and promote the recovery of patients in the treatment of acute bronchitis.

## 1. Introduction

Asthmatic bronchitis is a special kind of bronchitis, although its symptoms are basically similar to ordinary asthma symptoms, but this disease is more common in infants and young children; the disease symptoms are lung wheezing, breathing difficulties, chest tightness, phlegm, cough, wheezing, and so on [1]. Moreover, asthmatic bronchitis often occurs at night or in the morning, the onset is relatively slow, the course of the disease is long, and the repeated attacks of the child will promote the aggravation of the disease. If effective treatment is not taken in time, complications such as pneumonia and pulmonary heart disease can be triggered [2]. Pediatric asthmatic bronchitis is a bronchial infection in infants and young children with a complex pathogenesis that may be related to inflammatory cytokines and inflammatory mediators, such as neutrophils, lymphocytes, airway epithelial cells, interleukin-8 (IL-8), IL-10, and transforming growth *β* factor-beta (TGF-*β*). When the inflammatory response occurs in the bronchial airway, the airway is in a highly reactive state, coupled with a variety of external stimuli, the airway is blocked, the airflow is limited, and the child is easily accompanied by repeated episodes of wheezing [3].

Child-related suffering from a breathing disease swelling of the lung tubes is a sudden and severe swelling of the trachea related to the lung tubes mucosa caused by microbial infection and chemical stimulation or likely to have strong, bad body reaction factors. It is a common and often-happening disease in children, mostly secondary to upper breathing and lung-related area of land infections. Mainly, diseases that cause diseases include viruses, mycoplasma, dangerous lung disease, bacteria, or mixed infections [1]. Swelling of the lung tubes in infants and young children is called breathing loudly swelling of the lung tubes. Breathing disease signs of sickness appear in the early beginning and can be repeated, and the signs of sickness disappear when they reach school age. Bad skin redness, itching, and strong, bad body reactions of some people may develop related to lung tube breathing disease in old age [2]. Children suffering from a breathing disease swelling of the lung tubes and related to the lung tube breathing disease show the tube from the mouth to the lung hyperresponsiveness caused by breathing and lung-related area of land infection, and the basic disease-related changes are mainly crowding and blockage, swelling/fluid buildup, and insulting/swelling cell invasion at the infection site [3]. Through a series of reactions, bioactive substances are released, including blood-clotting fats. These are related to the lung tubes' smooth muscle contraction, mucosal crowding and blockage, and increased fluid release. Repeated events can lead to suffering from a breathing disease swelling of the lung tubes [4].

Now, people who work to find information often study or discuss the effects of traditional Chinese medicine in treating sicknesses from the parts of germ-killing, antiswelling, and harmful regulation. IFN*α*lb can directly reach the affected part of the breathing and lung-related area of land and increase the local drug concentration so that the drug effect can be quickly put into action, which can improve the following the law/doing as you are told of children and avoid the side effects caused by into the muscle injection happens [5]. Sang ju-Yin Decoction is a commonly used formula for children with cough and wind-heat disease. In vitro cell experiments show that it can stop nuclear-written version of spoken word factors and reduce the expression of insulting/swelling factors, which may be one of its antiswelling machines/methods [6]. HBD2 is one of the most studied germ-killing peptides. It has a certain relationship with breathing and lung-related sicknesses and has a certain germ-killing and bacteriostatic effect. Insulting/swelling factors (IL-lÎ^2^, etc.) can be written down through NF-KB nuclear-written version of spoken word factor channels, or other pathways cause increased expression [7]. There is no brought together as one end/end result on the role and legal/law-based machine/method/way of HBD2, and there are few medicine-based studies on its relationship with traditional Chinese medicine. Whether Sang ju-Yin Decoction can affect the expression of HBD2 by stopping insulting/swelling factors through a complex written version of spoken word channels is worth exploring [8]. Based on this, we have explored the effect of Sang ju-Yin Decoction combined with IFN*α*lb nebulization on children suffering from a breathing disease swelling of the lung tubes and the effects of IL-1*β* and HBD2. Now, the research results are reported as follows.

## 2. Material and Methods

### 2.1. Research Object

All records of patient identities included in this study will be kept at the hospital as required, and public reporting of study results will not disclose all records regarding patient identities. All patients gave informed consent before enrolling in the group; we fully communicated with patients before the experiment and introduced the experimental content and process, related risks, and possible adverse reactions; patients signed the informed consent form after obtaining the patient's consent; and we informed the patients of the test results in strict accordance with the experimental procedures. The clinical data of 80 cases of children with asthmatic bronchitis were selected as the object of this retrospective study, and they were divided into the control group and the observation group with 40 cases in each group according to different treatment methods. The general data such as gender and age of the patients in the two groups did not affect this trial, as shown in Table 1.

### 2.2. Exclusion Criteria

The inclusion criteria are as follows: (1) all patients in this study met the diagnostic criteria for pediatric asthmatic bronchitis in the “Guidelines for Primary Diagnosis and Treatment of Acute Tracheo-bronchitis (Practical Edition 2018)” [9]. (2) The disease duration of the patients was ≤3 weeks, and the body temperature was <38.5°C, with upper respiratory tract infection symptoms such as cough, expectoration, dry cough or a small amount of sputum, followed by mucopurulent sputum, increased sputum volume, aggravated cough, and occasionally blood in sputum can last 2-3 weeks, sometimes for several weeks. (3) The breath sounds of both lungs are coarse, and sometimes, wet rales can be heard. Most patients have normal chest X-ray examinations or thickened lung markings, and mycoplasma pneumonia IgM is positive (ELISA method). (4) All signed and agreed to the diagnosis and treatment plan. (5) Lastly are those who did not receive other treatment interventions.

The exclusion criteria are as follows: (1) patients with acute infectious diseases such as measles, whooping cough, influenza, malnutrition, and immunodeficiency and children who may seriously affect the self-limiting course of the disease and need to be excluded; (2) patients with severe heart, liver, kidney, digestion, and hematopoiesis and systemic and other serious primary diseases, those who cannot rule out cough caused by other diseases such as Mycobacterium tuberculosis infection, and those who are allergic to conventional therapeutic drugs or their components that need to be used during the test; (3) patients with allergic reactions or serious adverse events that occur during the test, the patient who suffers from other diseases, which affects the judgment of efficacy and safety, the test children who have poor compliance or request to withdraw from the clinical trial, and the test children who no longer receive a blood test; (4) patients who have been treated with hormones or other immunosuppressants; (5) patients with differences in treatment compliance; and (4) patients who stop the drug or give up treatment in the middle of the way.

## 3. Nursing Intervention Methods

Both groups of patients were given routine treatment, and the patients were instructed to rest more, eat a reasonable diet, drink more water, and change positions to promote the clearance of respiratory secretions. Symptomatic treatment of excessive sputum, asthma and allergies, oxygen if necessary, and anti-infective therapy if there is a bacterial infection. The control group was nebulized with IFN*α*lb. That is, budesonide and terbutaline were given through nebulized inhalation, and IFN*α*lb (20 *μ*g/piece, produced by Shenzhen Kexing Bioengineering Co. Ltd.) was added on the basis. The usage was IFN1 *μ*g/kg/day. It is divided into 2 atomized inhalations, and the course of treatment is 7 days. On the basis of the control group, the observation group was given Sang ju-Yin Decoction, that is, azithromycin dry suspension (100 g/bag; approved by Chinese medicine H10960112) (10 mg/kg), once a day. After three days of oral administration, the patients were stopped for four days. Seven days is the course of treatment, and the experimental course of treatment is 14 days (i.e., 2 courses of treatment). The addition or subtraction of Sang ju-Yin Decoction formula includes mulberry leaf 10 g, chrysanthemum 6 g, platycodon 8 g, almond 10 g, forsythia 6 g, Qianhu 8 g, tuckahoe 10 g, Fangfeng 6 g, Zhe Fritillaria 10 g, and licorice 3 g. Scutellaria 6 g was added for those with fever and, gypsum 15 g (decoction first) for sore throat; 10 g of a marigold root and 10 g of Scrophulariaceae were added; 10 g of bamboo rue and 10 g of loquat leaves with too much phlegm and yellow were added. First put the medicine in the container, add cold water over the medicine surface, soak for 30-60 minutes, and combine the medicines; each dose of Chinese herbal medicine is boiled with a strong fire. After boiling, use slow fire to maintain a slight boiling state, and continue to decoct for 15-20 minutes. Fry 100-200 mL and take it half an hour after meals (2 years old: 100 mL/day, divided into 2-3 times; 3-4 years old: 100-150 mL/day, divided into 2-3 times; and 5-14 years old: 150-200 mL/day, divided into 2-3 times). If the child's body temperature is greater than 38.5°C during the treatment process, physical cooling, antipyretic patches, and oral antipyretics (acetaminophen or ibuprofen) can be used for symptomatic treatment according to the situation.

## 4. Observation Indicators

### 4.1. Clinical Symptoms

The four typical clinical symptoms of asthmatic bronchitis in children, namely, cough, wheezing, pulmonary rales, and gas boosting, were scored, with 1-3 points for each item and 1-3 points for physical signs (the higher the score). It was indicated that the symptoms and signs are more severe.

### 4.2. Serum Indicators

For the children included in the trial, after signing the informed consent, 1 ml of whole blood was collected (using a sterile tube) before treatment (on the day of participating in the trial) and 14 days after treatment, and the blood was collected at 1000 × g centrifugation for 20 minutes; take the supernatant, aliquot, and freeze it in a -80°C refrigerator to detect IL-6 (ng/L), TNF-*α* (pg/L), IL-10 (ng/L), IL-1*β*, and HBD2. Respiratory frequency resistance (RR), tidal volume (TV), and peak expiratory flow (PEF) were measured by German SPIROSTIK spirometer before and after treatment.

## 5. Statistical Analysis

All statistical data in this study were entered into excel software by the first author and the corresponding author, respectively. The included data were tested by the Shapiro-Wilk method. The mean ± standard deviation (Mean ± SD) described the measurement data conforming to the normal distribution. The independent sample or paired-sample *t*-test was performed within the group, the count data were described by integer or percentage (%), and the *χ*^2^ test was used between or within the group. *M* (QR) described the included data that did not conform to the normal distribution, and the Mann–Whitney test was used, and the test level was *α* = 0.05.

## 6. Results

### 6.1. General Data Comparison

The difference in general clinical data such as gender, average age, course of disease, and body mass index showed no significant difference in general clinical data between the two groups (*P* > 0.05), and the two groups were comparable. See Table 1.

### 6.2. Comparison of Symptom and Sign Scores

There was no statistical difference in the scores of symptoms and signs between the two groups before treatment (*P* > 0.05), which was comparable, while the scores of shortness of breath, cough, stridor, lung rales, and signs after treatment were significantly different. And the observation group was lower than the control group, and the difference was statistically significant (*P* < 0.05). See Figure 1.

### 6.3. Comparison of Serum Inflammatory Markers

There was no significant difference in serum inflammatory indexes between the two groups before treatment (*P* > 0.05), while the differences in IL-6, IL-10, TNF-*α*, IL-1*β*, and HBD2 after treatment were significant, and the observation group was superior to the other. Compared with the control group, the comparison was statistically significant (*P* < 0.05). See Figure 2.

### 6.4. Comparison of Lung Function Indicators

The pulmonary function indexes of the two groups of patients were comparable before treatment (*P* > 0.05). After treatment, the RR, TV, and PEF indexes of the two groups of children were significantly improved. The RR and PEF of the observation group were lower than those of the control group, and the TV was higher than that of the control group. The comparison was statistically significant (*P* < 0.05). See Figure 3.

### 6.5. Adverse Reaction Comparison

After treatment, the adverse reaction rate of liver function damage, dry throat discomfort, rash, nausea and vomiting in the observation group was 7.5%, which was significantly lower than 27.5% in the control group, with statistical significance (*P* < 0.05). See Figure 4.

## 7. Discussion

IFN is highly related to living things' active glycoprotein, which is divided into two types according to its related to the body function of living thing features and activities. Among them, type I IFN includes IFN-a and type II IFN is IFN-y. Mononuclear macrophages mainly produce IFN-a. The main role in the disease-fighting system is a virus defense and device that controls something of people that ensures rules are followed [10]. Cells and fibroblasts can also make/create IFN*α*lb, which can directly resist viruses by causing some proteins, such as insulting/terrible protein kinase K, viral mRNA by 2,5 oligoadenylate synthase, and blocking viral protein translation. Through being unable to be harmed, regulation plays an indirect virus-killing role [11]. Therefore, the virus-killing effects and immunomodulatory effects of IFN provide related ideas about how things work or why they happen for effective treatment of suffering from a breathing disease swelling of the lung tubes [12]. Sang ju-Yin Decoction is a commonly used prescription for the medicine-based treatment of acute swelling of the lung tubes in children with wind-heat suddenly entering a place in an unwanted way the lung disease. Different doctors have their own, like nothing else in the world, understanding deep things and experience in the addition and subtraction of this prescription [13]. The addition and subtraction of Sang ju-Yin Decoction in this study are based on the addition and subtraction of Sang ju-Yin Decoction formula based on our many years of medicine-based experience (Zhejiang Fritillaria, licorice). This prescription has the functions of breaking up and moving away wind-heat, breaking up and moving away lung, resolving phlegm, and relieving cough, and it has the features of lightness and not coolness. It can get good results in medicine-based use. Therefore, scientific medicine-based instances of watching, noticing, or making a statement and research on the addition and subtraction of Sang ju-Yin Decoction prescription are carried out. It is of great importance and helps to summarize the experience of medicine-based effectiveness of traditional Chinese medicine [14].

In this study, the shortness of breath score, cough score, stridor score, lung rale score, and physical sign score of the two groups of patients after treatment were very different, and the instance of watching, noticing, or making a statement group was lower than the control group, pointing to that the addition or subtraction of Sang ju-Yin Decoction combined with IFN*α*lb Nebulization can improve signs of sickness and help increase in a good way the recovery of patients in the treatment of acute swelling of the lung tubes. Now, there is no specific treatment method for viral infection (showing signs of sickness), and supportive treatment methods are mostly used in medicine-based practice. In 1957, foreign-educated people discovered that IFN has broad-spectrum virus-killing effects and dual (related to the body function of living things) functions. On the one hand, it can stop virus reproduction without affecting (commonly and regular) cell functions [15]. On the other hand, it can control the inability to be harmed (harmful, angry behaviors) caused by breathing and lung-related virus infection, control the production of endogenous (able to be easily caught by others) poisonous chemicals, control the unable to be harmed function of the body, and improve the virus-killing effect [16]. The virus-killing (machine/method/way) of IFN is to directly limit the answer/copy and spread of the virus by binding to cell surface receptors, causing and activating virus-killing factors such as endogenous Mx protein and RNA-activating flowers; it can also directly or indirectly act on T cells and cells [17]. It controls the inability to be harmed response of the body, improves the phagocytic function of macrophages, helps increase/shows in a good way the production of (related to releasing a liquid) IgA in breathing and lung-related (related to sacs that surround body organs) cells, and improves local resistance. IFN has good virus-killing and immunomodulatory effects [18]. With the change for the better, over time of viruses, many viruses can block the signal transduction through receptors or otherwise interfere with the production of type I IFN, which can control the ability to be done and function of cells and affect the event of resistant cells [19]. Many previous studies have suggested that the addition of Sang ju-Yin Decoction or its combination therapy can improve the medicine-based effectiveness of cough, which may be related to the natural history of (suffering from a breathing disease) swelling of the lung tubes in children, because the self-healing ability of the disease needs/demands a certain amount of time and weeks The treatment time may cause the treatment difference between the experimental group and the control group to be unimportant [20]. Although there is no (a big change in numbers that means something important) difference between the addition and subtraction of Sang ju-Yin Decoction based on IFN*α*lb nebulization in terms of effectiveness or overall effectiveness (a process of figuring out the worth, amount, or quality of something), compared with simple western medicine treatment, both of them can accomplish or gain with effort higher effectiveness [21]. In terms of the complete disappearance time of cough, this study shows that the addition of Sang ju-Yin Decoction on the basis of IFN*α*lb (related to sprayed liquids) therapy can significantly shorten the cough disappearance time compared with the simple IFN*α*lb (related to sprayed liquids) treatment group [22].

In this study, the differences in IL-6, IL-10, TNF-*β*, IL-1*β*, and HBD2 after treatment were obvious, and the (instance of watching, noticing, or making a statement) group was better than the control group, pointing to/showing that the addition or subtraction of Sang ju-Yin Decoction has obvious effects and can reduce serum insulting/swelling index level. IL-6 can cause swelling response/angry responses, and its products come from various sources. A large number of experimental data show that IL-6 is an important proinsulting/swelling factor involved in different swelling responses/angry responses and sicknesses in the human body [23]. IL-6 can help increase/show in a good way the growing and spreading and using different things of inability to be harmed cells and improve their unable to be harmed function, and clearly connected or related research results show that with the improvement of human health, the expression level of IL-6 in the human body will decrease to a certain extent and slowly tend to be higher. Close to healthy levels, this is because IL-6 can activate T infection-fighting cells, cause the using different things of B infection-fighting cells, and finally release fluid immunoglobulin, which plays a role [24]. IL-10 is a multicellular and multifunctional cytokine, which is an essential human antiswelling factor, which can control human unable to be harmed function, control cell growth and using different things, and participate in human insulting and unable to be harmed responses. The medical community now recognizes it as insulting and reducing the body's ability to fight disease factors [25]. IL-10 is also an important disease-fighting system device that controls something/group of people that ensures rules are followed in the human body. It plays an important role in how a disease starts different sicknesses and is now recognized by the medical community as reducing the body's ability to fight disease factors [26]. IFN*α*lb is a multifunctional insulting/swelling cytokine, mainly produced by eosinophils and monocytes, with anti-infection and antitumor effects [27]. IFN*α*lb can help settle an argument the collection over time of eosinophils, infection-fighting cells, and eosinophils at the site of swelling, stimulate these cells to produce IL-6 and other factors, stop the cell death of eosinophils, and make mast cells and eosinophils. Endothelial fibroblasts or other organisms act as stimulators, causing the body to produce a swelling response that does not go away [28]. IFN*α*lb can help increase/show in a good way the release of fluid of Ig by stimulating the spread of B cells. In the body's swelling response/angry response, macrophages release a large amount of IFN*α*lb, which activates the surface stickiness/scar receptors of neutrophils and endothelial cells and helps increase/shows in a good way the release of insulting factors. TNF-*α* can affect the body's anti-infection ability. The worse the viral infection or bacterial infection, the higher the level of IFN*α*lb [29].

In this study, the RR, TV, and PEF indexes of the two groups of children were very much improved after treatment, and the RR and PEF of the instance of watching, noticing, or making a statement group were lower than those of the control group, and the TV was higher than that of the control group, showing that the addition or subtraction of Sang ju-Yin Decoction combined with IFN*α*lb nebulization can improve the effectiveness of the treatment. Improve the patient's lung function. Nebulization of IFN*α*lb can stimulate the contraction of a tube from the mouth to the lungs smooth muscle, stimulate the excretion of related to the lung tubes releases of fluid, reduce breathing and lung-related resistance, and secure/make sure of smooth breathing of patients. IFN*α*lb nebulization is a glucocorticoid with high antiswelling effect. The antiswelling effect can stop the release of active transmitters, such as something that triggers allergies and reduces the likelihood of having strong, bad body reactions. The addition or subtraction of Sang ju-Yin Decoction combined with IFN*α*lb nebulization significantly relieves medicine-based signs of sickness such as shortness of breath and breathing loudly and accomplishes or gains with an effort the purpose of very much improving lung-related fresh machines that bring fresh air function. The research results of foreign-educated people also support this view [30]. This study also found that the RR, PEF, and TV of instance of watching, noticing, or making a statement group improved more after treatment. It can be seen that the addition or subtraction of Sang ju-Yin Decoction combined with IFN*α*lb spraying into a mist has a cooperating effect. No serious bad reactions happened, and the two drugs were highly safe [31]. Although this study has some novelties, it also has faults/problems. It is more obvious to explore the medicine-based effect of adding or subtracting Sang ju-Yin Decoction and IFN*α*lb on children suffering from a breathing disease swelling of the lung tubes, but the clearly particular machine has not been deeply studied for a long time. The collected cases were from the same hospital, and the representativeness was poor, and both when something is kept out or not included and including in something were subject to some degree of judging things based on opinions and preferences instead of facts, which may lead to created unfair thinking in results. Moreover, the sample size is small, and the proportion of children with moderate and severe asthmatic bronchitis included is larger, resulting in a higher proportion of asthma developing, and the results may be biased. In the future, the sample size needs to be expanded to further explore the effect of modified Sang ju-Yin Decoction combined with interferon (IFN)*α*lb nebulization on children with asthmatic bronchitis and the effects of IL-1*β* and *β*-defensin 2 (HBD2).

## 8. Conclusion

In summary, the addition or subtraction of Sang ju-Yin Decoction combined with IFN*α*lb nebulization can improve signs of sickness and help increase in a good way the recovery of patients in the treatment of acute swelling of the lung tubes. The serum concentrations of IL-1*β* and HBD2 are related to the extreme harshness of suffering from a breathing disease swelling of the lung tubes in children. It can provide some reference for medicine-based treatment of suffering from a breathing disease swelling of the lung tubes in children.

## Figures and Tables

**Figure 1:** Comparison of symptom and sign scores. According to the test standard of *α* = 0.05, the shortness of breath score (a), cough score (b), stridor score (c), and lung rale score (d) after treatment in the two groups and sign score (e) were significantly improved, and the symptom and sign score of the observation group was significantly lower than that of the control group. Values are expressed as the mean ± standard deviation and analyzed by an independent samples *t*-test. After treatment, the shortness of breath score, cough score, stridor score, lung rale score, and physical sign score of the observation group were lower than those of the control group (*P* < 0.05).

**Figure 2:** Comparison of serum inflammatory markers. The comparison of serum inflammatory indexes before treatment was analyzed by independent samples *t*-test (*P* > 0.05). After treatment, the levels of IL-6 (Figure 3(a)), IL-10 (Figure 3(b)), TNF-*α* (Figure 3(c)), IL-1*β* (Figure 3(d)), and HBD2 (Figure 3(c)) in the observation group were higher than those of the control group. According to the test standard of *α* = 0.05, the value is expressed as the Mean ± SD, indicating that the independent samples *t*-test was used for analysis, and the differences in IL-6, IL-10, TNF-*α*, IL-1*β*, and HBD2 after treatment were obvious, and the observation group was superior to the other. In the control group, *P* < 0.05.

**Figure 3:** Comparison of pulmonary function indicators. The pulmonary function indexes of the two groups before treatment were comparable, and the independent samples *t*-test was used for analysis (*P* > 0.05). After treatment, the RR (a) and PEF (c) of the observation group were lower than those of the control group, and the TV (b) was higher than that of the control group. According to the test standard of *α* = 0.05, the value is expressed as the Mean ± SD, which means that the independent samples *t*-test was used for analysis. The RR and PEF of the observation group were lower than those of the control group, and the TV was higher than that of the control group (*P* < 0.05).

**Figure 4:** Comparison of adverse reactions. After treatment, the adverse reactions of the two groups were significantly improved, and the self-protection ability score of the observation group was significantly higher than that of the control group. According to the test standard of *α* = 0.05, the value is expressed as an integer, and the chi-square test is used for analysis. The adverse reaction rate of liver function damage, dry throat, rash, nausea, and vomiting was 7.5%, which was significantly lower than 27.5% of the control group (*P* < 0.05).

**Table 1:** Comparison of general data between the two groups (*n*, $\bar{x}\pm \text{s}$).

Group	Gender (men/women)	Average age (age)	Course of disease (week)	Body mass index (kg/m^2^)
Comparison group (40)	18/22	3.50 ± 1.32	5.6(3.7~7.9)	27.78 ± 2.32
Observation group (40)	17/23	3.69 ± 1.66	5.5(3.1~7.7)	27.62 ± 2.66
*χ* ^2^/*t*	0.051	-0.567	0.040	0.020
*P*	0.822	0.573	0.965	0.984

## Data Availability

No data were used to support this study.

## References

[1] Morice A. H., Millqvist E., Bieksiene K. (2020). ERS guidelines on the diagnosis and treatment of chronic cough in adults and children. *The European Respiratory Journal*.

[2] Cheng C., Zou G. S., Lin H. Q. (2020). Inhalation of budesonide suspension combined with compound ipratropium bromide aerosol for the treatment of asthmatic bronchitis in children. *Shenzhen Journal of Integrated Traditional Chinese and Western Medicine*.

[3] Hong J., Lou S. Z., Wang P. (2019). Analysis of 45 cases of asthmatic bronchitis in children treated with the combination of salbutamol nebulized inhalation. *Chinese Journal of Critical Care Medicine*.

[4] Ruffles T. J. C., Marchant J. M., Masters I. B. (2021). Outcomes of protracted bacterial bronchitis in children: a 5-year prospective cohort study. *Respirology*.

[5] Li Y., Williams R. J., Dombrowski N. D. (2020). Current evaluation and management of plastic bronchitis in the pediatric population. *International Journal of Pediatric Otorhinolaryngology*.

[6] Kallam E. F., Kasi A. S., Patki R. (2021). Bronchoscopic interventions for plastic bronchitis in children without structural heart disease. *European Journal of Pediatrics*.

[7] Weinberger M., Hurvitz M. (2020). Diagnosis and management of chronic cough: similarities and differences between children and adults. *F1000Research*.

[8] Michalska A., Blaszczyk K., Wesoly J., Bluyssen H. A. R. (2018). A positive feedback amplifier circuit that regulates interferon (IFN)-stimulated gene expression and controls type I and type II IFN responses. *Frontiers in Immunology*.

[9] Traditional Z. P., Medicine C., Therapy F. (2016). Hypertension control: a narrative review of Chinese literature. *The American Journal of Chinese Medicine*.

[10] Yu Q., Chen W., Zhong J., Qing D., Yan C. (2021). Structural elucidation of three novel oligosaccharides from Kunlun Chrysanthemum flower tea and their bioactivities. *Food and Chemical Toxicology*.

[11] Yan H. Y., Liu Y., Xu Y., Fang Y., Guo L. P., Liu D. H. (2021). Analysis and evaluation of mineral elements of Chrysanthemum morifolium for medicinal and tea use of different germplasm resources. *Zhongguo Zhong Yao Za Zhi*.

[12] Chinese Medical Association (2019). Guidelines for primary diagnosis and treatment of respiratory system diseases writing expert group. Guidelines for primary diagnosis and treatment of acute tracheo-bronchitis (practice version 2018). *Chinese Journal of General Practitioners*.

[13] Medina G. N., de Los S. T., Diaz-San S. F. (2020). Use of IFN-based biotherapeutics to harness the host against foot-and-mouth disease. *Frontiers in Veterinary Science*.

[14] Zanoni I., Granucci F., Broggi A. (2017). Interferon (IFN)-*λ* takes the helm: immunomodulatory roles of type III IFNs. *Frontiers in Immunology*.

[15] van de Vosse E., van Dissel J. T. (2017). IFN-*γ*R1 defects: mutation update and description of the IFNGR1 variation database. *Human Mutation*.

[16] Chen L., Liu Y., Huang X. (2021). Comparison of chemical constituents and pharmacological effects of different varieties of Chrysanthemum Flos in China. *Chemistry & Biodiversity*.

[17] Chen B. Y., Liao J. H., Hsu A. W., Tsai P. W., Hsueh C. C. (2018). Exploring optimal supplement strategy of medicinal herbs and tea extracts for bioelectricity generation in microbial fuel cells. *Bioresource Technology*.

[18] Karimi Y., Giles E. C., Vahedi F. (2020). IFN-*β* signalling regulates RAW 264.7 macrophage activation, cytokine production, and killing activity. *Innate Immunity*.

[19] Li Q., Zhou Y., He W. (2021). Platelet-armored nanoplatform to harmonize janus-faced IFN-*γ* against tumor recurrence and metastasis. *Journal of Controlled Release*.

[20] Úsuga-Monroy C., González Herrera L. G., Echeverri Zuluaga J. J., Díaz F. J., López-Herrera A. (2020). IFN-*γ* mRNA expression is lower in Holstein cows infected with bovine leukemia virus with high proviral load and persistent lymphocytosis. *Acta Virologica*.

[21] Li J., Zeng M., Yan K., Yang Y., Li H., Xu X. (2020). IL-17 promotes hepatocellular carcinoma through inhibiting apoptosis induced by IFN-*γ*. *Biochemical and Biophysical Research Communications*.

[22] Hu Y., Alnabulsi A., Alnabulsi A. (2021). Characterisation and analysis of IFN-gamma producing cells in rainbow trout Oncorhynchus mykiss. *Fish & Shellfish Immunology*.

[23] Kim A. R., Kim H. S., Kim D. K. (2016). The extract of Chrysanthemum zawadskii var. latilobum ameliorates collagen-induced arthritis in mice. *Evidence-Based Complementary and Alternative Medicine*.

[24] Hong S. I., Kwon S. H., Kim M. J. (2012). Anxiolytic-like effects of Chrysanthemum indicum aqueous extract in mice: possible involvement of GABAA receptors and 5-HT1A receptors. *Biomolecules & Therapeutics*.

[25] Chen L. X., Hu D. J., Lam S. C. (2016). Comparison of antioxidant activities of different parts from snow chrysanthemum (Coreopsis tinctoria Nutt.) and identification of their natural antioxidants using high performance liquid chromatography coupled with diode array detection and mass spectrometry and 2, 2′-azinobis (3-ethylbenzthiazoline-sulfonic acid) diammonium salt-based assay. *Journal of Chromatography A*.

[26] Shon J. C., Kim W. C., Ryu R. (2020). Plasma lipidomics reveals insights into anti-obesity effect of Chrysanthemum morifolium ramat leaves and its constituent luteolin in high-fat diet-induced dyslipidemic mice. *Nutrients*.

[27] Gregory M. A., Manuel-Apolinar L., Sánchez-Garcia S. (2019). Soluble intercellular adhesion molecule-1 (IL-1*β*) as a biomarker of vascular cognitive impairment in older adults. *Dementia and Geriatric Cognitive Disorders*.

[28] Hoxha M., Rovati G. E., Cavanillas A. B. (2017). The leukotriene receptor antagonist montelukast and its possible role in the cardiovascular field. *European Journal of Clinical Pharmacology*.

[29] Horiuchi T., Mitoma H., Harashima S., Tsukamoto H., Shimoda T. (2010). Transmembrane TNF-alpha: structure, function and interaction with anti-TNF agents. *Rheumatology (Oxford, England)*.

[30] Godfrey M. S., Friedman L. N. (2019). Tuberculosis and biologic therapies: anti-tumor necrosis factor-*α* and beyond. *Clinics in Chest Medicine*.

[31] Cruceriu D., Baldasici O., Balacescu O., Berindan-Neagoe I. (2020). The dual role of tumor necrosis factor-alpha (TNF-*α*) in breast cancer: molecular insights and therapeutic approaches. *Cellular Oncology*.

